The article "Prokineticins as a Prognostic Biomarker for Low-Grade Gliomas: A Study Based on The Cancer Genome Atlas Data" was retracted in 2024. Reasons: signs of a paper mill; suspected computer-generated content; unreliable results or conclusions; concerns about the data.

# Prokineticins as a Prognostic Biomarker for Low-Grade Gliomas: A Study Based on The Cancer Genome Atlas Data

**DOI:** 10.1155/2022/2309339

**Published:** 2022-07-07

**Authors:** Junqing Zhong, Ding Xiang, Xinlong Ma

**Affiliations:** ^1^Department of Rehabilitation, Tianjin Hospital, Tianjin, China; ^2^Department of Orthopedics, Tianjin Hospital, Tianjin, China

## Abstract

Lower-grade glioma (LGG) is a crucial pathological type of glioma. Prokineticins have not been reported in LGG. Prokineticins as a member of the multifunctional chemokine-like peptide family are divided into two ligands: PROK1 and PROK2. We evaluated the role of PROK1 and PROK2 in LGG using TCGA database. We downloaded the datasets of LGG from TCGA and evaluated the influence of prokineticins on LGG survival by survival module. Correlations between clinical information and prokineticins expression were analyzed using logistic regression. Univariable survival and multivariate Cox analysis was used to compare several clinical characteristics with survival. Correlation between prokineticins and cancer immune infiltrates was explored using CIBERSORT and correlation module of GEPIA. We analyzed genes of PROK1 and PROK2 affecting LGG, screened differentially expressed genes (DEGs), interacted protein-protein with DEGs through the STRING website, then imported the results into the Cytospace software, and calculated the hub genes. To analyze whether hub genes and prokineticins are related, the relationship between PROK1 and PROK2 and hub genes was assessed and shown by heat map. In addition, gene set enrichment analysis (GSEA) was performed using the TCGA dataset. The univariate analysis using logistic regression and PROK1 and PROK2 showed opposite expression differences between tumor and normal tissues (*p* < 0.05). PRO1 and PROK2 expressions showed significant differences in tumor grade, age, Iiscitrate DeHydrogenase (IDH) status, histological type, and 1P/19q codeletion. Multivariate analysis revealed that the up-regulated PROK1 and PROK2 expression is an independent prognostic factor for bad prognosis. Specifically, prokineticin expression level has significant correlations with infiltrating levels of Th1 cells, NK CD 56bright cells, and Mast cells in LGG. We screened 21 DEGs and obtained 5 hub genes (*HOXC10*, *HOXD13*, *SOX4*, *GATA4*, *HOXA9*). GSEA-identified FCMR activation, creation of C4 and C2 activators, and CD22-mediated BCR regulation in gene ontology (GO) were differentially enriched in high PROK1 and PROK2 expression phenotype pathway, cytoplasmic ribosomal proteins, and ribosome and were differentially enriched in the low PROK1 and PROK2 expression phenotype pathway. Prokineticins are a prognostic biomarker and the correlation between hub genes and LGG requires further attention.

## 1. Introduction

Low-grade gliomas (LGG), also known as grade I and grade II gliomas, originate from the glial cells of the primary slow-growing brain tumors and account for approximately15% of all primary brain tumors [1]. LGG is the most common invasive tumor in the adult cerebral hemisphere, including astrocytoma, oligodendrocyte, and astrocytoma, and is most common in young people under 50 [2]. Because of its highly diffuse nature, complete neurosurgical resection is challenging, and residual tumors can lead to recurrence and higher levels of progression [3]. At present, WHO's histologic classification is still used in LGG classification, but the clinical treatment plan is influenced by image examination, histological classification, and WHO classification.

There has been considerable debate about the best treatment strategy for LGG [4], such as surgery, chemotherapy, and radiation therapy. However, recent studies have found that the prognosis of LGG is inconsistent with WHO classification, and clinical decision-making may be better guided by genetic classification. Clinicians and scientists have delved into identifying molecular markers associated with gliomas and pathology that influences a patient's individualized treatment [5]. We aim to accurately predict patient survival or response to individualized therapy; new biomarkers were identified in patients with gliomas.

Prokineticins belong to a family of multifunctional chemokine-like peptides and were identified forty years ago [6]. The researchers identified two phenotypes, PROK1 and PROK2 [7], based on the homology of human protein codes (proteins isolated from the dendroaspis polylepis venom [8] and skin secretions of bomtina variegat [6]). Numerous studies have found that prokineticins and their receptors are found in various human tissues, such as the brain, heart, bone marrow, and peripheral blood. Since they are distributed in different cells and tissues and exhibit a wide range of tissue-specific biological activities, they coordinate complex behaviors, such as feeding, circadian rhythms, and hyperalgesia [9]. They are further involved in neuronal migration [10], survival, angiogenesis, hematopoiesis, and inflammation.

Prokineticins have been detected in the central nervous system [11], anterior horn of the spinal cord [12], and other nerve tissues for 20 years. Prokineticins can be tissue-specific cell survival factors regulating LGG, and their ability to induce angiogenesis and coordinate inflammatory immune responses has got our attention. Therefore, we used LGG-related data from The Cancer Genome Atlas (TCGA) to determine the correlation between prokineticins and LGG using R and Gene Expression Profiling Interactive Analysis (GEPIA). In addition, we detected the correlation between the expression of kinetin and density of tumor infiltrating immune cells (TIICs) in different tumor microenvironments. We screened the differentially expressed genes (DEGs) in LGG for up- and down-regulated hub genes that may be relevant targets or biomarkers and contribute to the potential positive role of prokineticins in LGG.

## 2. Materials and Methods

### 2.1. Data Acquisition

Level 3 HTSeq-FPKM RNAseq datasets from the LGG project were selected from the Open TCGA database (https://portal.gdc.cancer.gov/) [13]. The RNAseq data obtained in the fragments per kilobase per million (FPKM) format was converted to Transcripts Per Million reads (TPM) format and Log2 converted to eliminate the control/normal missing entries. Based on the expression of PROK1 and PROK2, the tumor tissues were divided into two groups: low expression group, 0–50%; high expression group, 50–100%.

### 2.2. Expression and Survival Analysis of PROK1 and PROK2

The correlation between the expression of PROKR1 and PROK2 in LGG and the clinicopathological information was confirmed online from the GEPIA database (http://GEPIA.cancer-pku.cn/index.html) [14]. A box map was constructed according to the disease status (tumor or normal), and the differential expression of PROK1 and PROK2 was calculated. GEPIA database integrates TCGA big data, for cancerous tissue, and GTEx big data, for normal tissue, and uses bioinformatics to answer important questions in cancer pathophysiology; reveal cancer subtypes; drive the expression of genes, alleles, and differentially expressed or carcinogenic factors; and explore new cancer targets and markers.

The main clinical parameters of PROK1 and PROK2, expression, grade, gender, age, IDH status, histological type, and 1p/19q were statistically analyzed using R (3.6.3); ggplot2 was used for visual rendering [15].

### 2.3. Detection of TIICs Immune Response in LGG

CIBERSORT (http://cibersort.stanford.edu/) is a deconvolution algorithm based on gene expression used to evaluate the relative changes in the expression of a group of genes in a sample [16]. We used CIBERSORT to measure the immune responses of 21 kinds of TIICs in LGG and evaluated the correlation between survival rate and molecular subsets. By establishing the gene expression dataset using standard annotation files, the algorithm is uploaded to the CIBERSORT website, and the algorithm runs with a default signature matrix of 1000 permutations. CIBERSORT estimated the *P* value of deconvolution by Monte Carlo sampling and determined the confidence of the results. We used 529 LGG samples from TCGA, and low expression and high expression groups each accounted for 50% of the samples; furthermore, we used the GSVA package in R (3.6.3) for vioplot [17].

### 2.4. Differential Expression Analysis of PROK1 and PROK2 in Pan Cancer

We analyzed the expression differences of PROK1 and PROK2 using the Level 3HTSeq-FPKM data of the Universal Cancer Project in TCGA database, the RNAseq data in FPKM format is converted to log2, and the result is visualized.

### 2.5. Analysis of Differentially Expressed Genes(DEGs)

Using R, we analyzed the RNAseq data of PROK1 and PROK2 for LGG obtained from the TCGA database and found that the screening criteria met | log2(FC) | >1.5 and *p*. adj<0.05, and Venn set, PROK1 and PROK2 common DEGs were obtained. The results (DEGs) were imported into the STRING online site [18], where protein-protein interactions (PPI) were used to obtain the intergenic network of DEGs and then imported into Cytospace [19]. The DEGs were calculated from node to node using the cytoHubba plug-in on the Cytospace [20]; the top 5 hub genes were selected according to “Degree.” The selected hub gene and PROK1 and PROK2 were analyzed and validated the correlation by the molecular heat map. The groups were classified according to 50% of the low- and high-expression groups.

### 2.6. Gene Enrichment Analysis

For gene enrichment analysis, we used the gene set enrichment analysis (GSEA) method [21], which uses a predefined set of genes and sorts them according to their expression in the two types of samples. In this study, GSEA generated an initial list of gene classifications based on its association with the expression of PROK1 and PROK2. This calculation illustrates the differences between the high and low expression of PROK1 and PROK2 groups. For each analysis, we performed 1000 repeated gene set permutations and presented the phenotypic labels for the expression of PROK1 and PROK2. In addition, we used the *P* values, normalized enrichment score (NES), and false discovery rate (FDR) <0.05, as criteria for selecting and classifying significant enrichment outcomes in each phenotype [22].

### 2.7. Statistical Analysis

The data obtained from TCGA were analyzed using R (3.6.3). The Shapiro-Wilk normality test was used to analyze PROK1 and PROK2 data, and the Pearson correlation coefficient was used to transform the unsatisfied variables [23]. The Wilcoxon rank sum test was used to compare the expression of PROK1 and PROK2 between variations in clinical parameters (tumor, grade, gender, age, IDH status, and histological type) [24]. Using the Shapiro-Wilk normality test for 21 kinds of TIICs, the Wilcoxon sum test or analysis of variance was used to determine whether it was in accordance with the normal distribution (the results showed significant difference if *P* < 0.05. Marked by: ns, *P* ≥ 0.05; ∗, *P* < 0.05; ∗∗, *P* < 0.01; ∗∗∗, *P* < 0.001).

## 3. Results

### 3.1. Characteristics and Multifactorial Analysis of Patients

In October 2021, clinical and gene expression data of 529 patients with LGG were obtained on the TCGA website, excluding the cases with insufficient or missing data on age and total survival time. We analyzed the effect of low and high expression of PROK1 and PROK2 on the median sex and age of WHO Grade and Gender, respectively, as shown in Table 1. In addition, the Pearson correlation analysis was used to determine the correlation between PROK1 and PROK2. The results showed that there was a positive correlation between PROK1 and PROK2 (*R* =0.11, 95% CI =0.029-0.197, *P* = 0.009), as shown in Figure 1. The area of PROK1 and Prok2 was close to each other. The sensitivity of PROK1 and PROK2 was 0.711 (cut-off 0.328) and 0.824, respectively. The negative predictive value for both PROK1 and PROK2 was more than 0.8, as shown in Figure 2.

### 3.2. Survival Analysis and Clinical Multifactorial Expression of PROK1 and PROK2

The survival curve and expression boxmap of normal and tumor tissues were constructed using GEPIA analysis, as shown in Figure 3. The results showed that PROK1 and PROK2 were significantly correlated with overall survival in different states (*P* < 0.01). In addition, the expression of PROK1 in tumor tissue samples was significantly higher than that in normal tissue samples (*P* < 0.05), as shown in Figure 3(a1); the expression of PROK2 in tumor tissue samples was significantly lower than that in normal tissue samples (P <0.01), as shown in Figure 3(b1). The median survival time of low and high expressions of PROK1 was 135.6 and 63, respectively (P =0.028), as shown in Figure 3(a2), and the median survival time of low and high concentrations of PROK2 was 95.8 and 51.6, respectively (P =0.008), as shown in Figure 3(b2).

According to Figure 4(a), the expression of PROK1 is more significant than that of PROK2 (median 0.847 : 0.184). With the progression of grade, although the expression of PROK1 significantly increased (*P* = 0.003), the expression of PROK2 was not significantly different (*P* = 0.989), as shown in Figure 4(b). We compared the variation in high and low expressions as per sex, age, IDH status, histological type, and 1p/19q co-deletion; the results are shown in Figures 4(c)–4(g). The expression of PROK1 in grade (*P* = 0.003) and age (*P* = 0.005) was significant, while the expression of PROK2 in IDH status (*P* < 0.001) and 1p/19q co-deletion (*P* = 0.007) was significant. Multivariate Cox analysis showed that tumor grade, age, IDH status, 1p/19q co-deletion, and PROK1 and PROK2 were multivariate Cox analysis of forest plot for LGG, as shown in Figure 5.

### 3.3. Expression of PROK1 and PROK2 in TIICs

Azimi et al. have shown that lymphocyte is an independent predictor of sentinel lymph node status and survival in cancer patients [25]. Based on this theory, we hypothesized that the expression of PROK1 and PROK2 was related to the immunologic invasion of LGG. A total of 529 tumor specimens were divided into two groups based on PROK1 and PROK2 expression.  Figure 6 shows the proportion of 21 immune cell subsets in which Th1 cells, CD56 bright NK cells, and mast cells were the main immune cells affected by the expression of PROK1 and PROK2. Interestingly, the high and low expression of PROK1 and PROK2 had the opposite effect on Th1 cells (*P*^PROK1^0.001: *P*^PROK2^0.000). Except for the immune cells affected by Th1 cells, CD56 dim NK cells, neutrophils, macrophages, eosinophils, cytotoxic cells, and B cells, there were significant differences in the expression of PROK2 (*P* < 0.001), while the expression of PROK1 had relatively little effect on immune cells (TFH).

### 3.4. Differential Analysis of Pan Cancer

A total of 11,093 samples (para 730: tumor 10363) were obtained from the TCGA database. The expressions of PROK1 and PROK2 in 33 kinds of Pan cancer were analyzed. In addition to LGG, the expressions of PROK1 in BLCA, BRCA, COAD, HNSC, KICH, KIRP, and PRAD in tumor group were significantly lower than those in normal group (*P* < 0.001). The expression of PROK2 in BRCA, LIHC, LUAD, LUSC, and UCEC in tumor group was significantly lower than that in para-cancer group (*P* < 0.001) (Figure 7).

### 3.5. Comparison of DEGs of PROK1 and PROK2 in LGG and Screening of Hub Genes

The screening condition for the differential genes was to satisfy the | log2(FC) | >1.5 and *p*. adj<0.05 criteria. Among those that satisfied the criteria, 50 differentially expressed genes were obtained from PROK1, 45 were up-regulated and 5 were down-regulated, and 348 were obtained from PROK2, 345 were up-regulated and 3 were down-regulated. A Venn map was constructed by crossing the PROK1 and PROK2, and a total of 21 DEGs were obtained (Figure 8(a)), which were imported into the STRING protein-protein interaction database. The results were screened for hub genes using the cytoHubba plug-in in Cytospace; *HOXC10*, *HOXD13*, and *SOX4* were selected according to “Degree”; *GATA4* and *HOXA9* are the hub genes of PROK1 and PROK2, in which *SOX4* is the down-regulated gene and the rest is the up-regulated gene (Figure 8(b)).

To verify whether there were significant differences among the five hub genes screened by Cytospace, we performed a Pearson coefficient analysis of them, as shown in Table 2. We found that, except for the nonsignificant correlation between GATA4 and PROK1, the remaining hub genes were significantly different for PROK1 (Figure 9(a)) and PROK2 (Figure 9(b)) and were visualized with heat map.

### 3.6. Enrichment Analysis of Prokineticins

Based on the GSEA signal pathway to identify correlations between different expression datasets of PROK1 and PROK2 in LGG, five high and low expression enrichment pathways of PROK1 (Figures 10(a) and 10(b)) and PROK2 (Figures 10(c) and (d)) have been listed, respectively, by NRS. Activation of FCGR, creation of C4 and C2 activators, and regulation of CD22-mediated BCR were observed in PROK1 and PROK2. Further, cytoplasmic ribosomal proteins and ribosome were detected in PROK1 and PROK2.

## 4. Discussion

Little is known about the role of prokineticins in human cancer, and current research is only related to the pathogenesis of a few cancers [26, 27]. Studies revealed that prokineticins have similar affinity to two homologous 7-transmembrane g protein-coupled receptors (PROKR1 and PROKR2). Prokineticins are highly conserved among species and are characterized by N-terminal AVIT consensus sequence and 5-disulfide bonds [28]. Prokineticins and their receptors are distributed in various human tissues, such as the ovaries, testes, adrenal glands, brain, heart, and bone marrow. They show a wide range of tissue-specific biological activities [9]. They coordinate complex behaviors, such as eating, drinking, circadian rhythm, and hyperalgesia, and also participate in neuron migration and survival, angiogenesis, hematopoiesis, and inflammation [29]. This diversity stems from the difference in their distribution in tissues. Their receptors can activate a variety of signaling events. In different tissues, the expression of PROK1 is significantly different from that of human multiple myeloma cells. In hepatocellular carcinoma, the expression of PROK2 is inversely proportional to the degree of malignancy; although the two have similar homology, their differences exist in a wide range of tissue-specific biological activities. In view of their role in tumor pathophysiology, as survival factors of some tissue-specific cells, their ability to induce angiogenesis and coordinate proinflammatory immune response may be one of the major causes of cancer.

We found that changes in the expression of PROK1 and PROK2 were closely related to the prognosis of LGG; their expression is inversely proportional to the prognosis. Downregulation of their expression is an independent prognostic factor indicating a positive prognosis. Xiao et al. [30] showed that PROK1 was overexpressed in human glioma, but not in normal human brain tissue, and the expression was proportional to WHO grade, which was consistent with our study. Therefore, the prognosis of high expression of PROK1 with a value of LGG was poor. In addition, our research showed that different immune marker sets and immune infiltration levels were related to the expression of PROK1 and PROK2 in LGG. Therefore, PROK1 and PROK2 may influence tumor immunology and be potential tumor biomarkers. In this study, we observed that there were significant differences in the expression of PROK1 and PROK2 in normal and LGG tissues. To further study the potential mechanism underlying the expression of prokineticins in cancer, we downloaded the dataset from TCGA. TCGA analysis using R(3.6.3) showed that the expression of PROK1 and PROK2 was related to tumor grade. Multivariate analysis showed that the expression of PROK1 and PROK2 was an independent factor influencing the prognosis of a patient with LGG. Clinical data showed that PROK1 was closely related to age; PROK2 was significantly different from IDH status, and its expression was higher in WT. In addition to comparing the expression of LGG, we also performed extended analysis of the expression of Pan in order to find out whether PROK1 and PROK2 are similar to LGG in other cancers, and we found that there were significant differences in the expression of Pan cancer and adjacent tissues, which confirmed that there were co-expression in different tissues, but there were significant differences in expression pattern [31]. The high and low expression of PROK2 was significantly different in the analysis of immunologic infiltration (Th1, NK CD56dim, NK CD56bright, Neutrophil, Mast, Macrophages, Eosinophils, Cytotoxic, and B-cells); previous studies have also shown that PROK2 limited the expression of natural immune cells, such as neutrophil, monocytes, and macrophages. Zhong et al. [32] studied that PROK2 promotes the mobilization of hematopoietic cells and neutrophil chemotaxis and triggers the release of proinflammatory cytokine from bone marrow cells, whereas PROK1 is less expressed in immune cells, but it can regulate the differentiation and activation of monocytes [27]. Our analysis showed that the expression of PROK1 and PROK2 is significantly related to TH1 cells, NK CD56 bright cells, and master cells in LGG, suggesting PROK1 and PROK2 are of great significance in regulating the immune microenvironment in LGG tumors. We found that the high expression of PROK1 and low expression of PROK2 were significantly different for Th1 cells. Therefore, there may be a correlation between the changes in expression of the two ligands in LGG. According to Montfort et al., the expression of immune characteristics among different immune cell types is closely related, indicating diverse, predictable, and consistent immune infiltration in tumor conditions. Therefore, the influence of PROK1 and PROK2 on LGG may be related to T cells, NK cells, and B cells. Central nervous system tumors show a strong dependence on glycolysis [33], so a ketosomal diet has become an important tool in the treatment of brain gliomas; the mechanism may be through enhancing antitumor immunity and changing gene expression to improve the sensitivity of weight-bearing chemotherapy and then affect the growth of tumor.

To understand the differential gene expression of PROK1 and PROK2 in LGG, we imported the screened differential genes into Cytospace, based on the results of online PPI analysis using data from STRING, obtained the five most significant hub genes through “Degree,” and verified the five hub genes by the Pearson correlation analysis. Except for *GATA4*, there was no significant difference in PROK1. Among them, *HOXC10*, *HOXD13*, and *HOXA9* are homeobox family of genes, which play an important role in the morphogenesis of multicellular organisms [34]. *HOXC10* is closely related to EGFR (Epidermal Growth Factor Receptor). *EGFR* is closely related to tumor cell proliferation, invasion, and angiogenesis, *EGFR* may also be involved in tumor angiogenesis, and in the highly vascularized LGG, the *EGFR* promoter may be involved in inducing angiogenesis and thus accelerating tumor cell proliferation and invasion. Curtis et al. [35] used an antagonist called PROK2 to reduce the branching of endothelial cells. Interestingly, in previous studies, a protein called endocrine gland-derived vascular endothelial growth factor (EGVEGF) was highly homologous to PROK1 [31]. EGVEFG and EGFR are of the same vascular endothelial growth factor, both of which promote angiogenesis, which may be one of the reasons that PROK1 expression is proportional to the malignant degree of LGG. *SOX4*, a member of the *SOX* family and no introns, combines with other proteins to form a complex and can be a transcription regulatory factor, which mediates the apoptosis of cells and tumors. The study found that SOX4 is closely related to the invasion and specialization of various tumors [36, 37], and Lin et al. [38] have previously found that SOX4 is more expressed in gliomas, which may be related to its role in the central nervous system development. PROK1 and PROK2 not only affect LGG through immune cells but also indirectly affect the expression of genes of LGG and the occurrence and development of this tumor through multiple genes [39].

To further study the functions of prokineticins in LGG, we used TCGA data to conduct GSEA, which showed CD22-mediated BCR regulation. Creation of C4 and C2 activators and activation of FCGR are differentially enriched in PROK1 and PROK2 high expression phenotypes and in ribozyme and cytogenetic fundamental proteins in PROK1 and PROK2 low expression phenotypes. The concentration changes of PROK1 and PROK2 can activate FCGR, which acts on complement and B cells and cell ribosomes. The participation and signal activity of FCGR can further stimulate different types of immune cells, such as DC, macrophages, or neutrophils, and further change the adaptive immune response through antigen presentation, cytokine production, and chemotaxis. Therefore, prokineticins can be potential indicators of LGG prognosis and act as therapeutic targets.

## 5. Conclusion

Prokineticins may be potential molecular markers that will aid in predicting the prognosis of patients with LGG. In addition, the possible key pathway underlying prognosis is regulated by PROK1 and PROK2 through ribosomes and by activating FCGR. We suggest further research on this topic, especially on hub genes, to improve the evidence on the biological effects of prokineticins.

## Figures and Tables

**Figure 1:** PROK1 and PROK2 correlation analysis. Pearson correlation coefficient r =0.110, *P* =0.009, indicating that there is a positive correlation between PROK1 and PROK2.

**Figure 2:** ROC of PROK1 and PROK2. The area under the ROC curve of PROK1 and PROK2 is 0.766 and 0.738, respectively. The cut-off value, sensitivity, specificity, positive predictive value, negative predictive value, and Yoden index of PROK1 were 0.328, 0.711, 0.694, 0.514, 0.841 and PROK2 were 0.104, 0.558, 0.824, 0.590, 0.804, and 0.382, respectively.

**Figure 3:** The survival curve and expression boxmap of normal and tumor tissues were constructed using GEPIA analysis. (a1) Comparison of PROK1 expression between normal and tumor tissues. (b1) Comparison of PROK2 expression between normal and tumor tissue. In PROK1, tumor group was higher than normal group; the difference was statistically significant (*P* < 0.05). In PROK2, tumor group was lower than normal group; the difference was statistically significant (*P* < 0.01). (a2) The survival curve of low and high concentration PROK1 was compared (*P* = 0.028). (b2) The survival curve of low and high concentration PROK2 was compared (*P* = 0.008). The concentrations of PROK1 and PROK2 had significant difference for survival.

**Figure 4:** Clinical multifactorial expression of PROK1 and PROK2. (a) Expression of PROK1 and PROK2 in tumor tissue. (b) Expression of low and high concentrations of PROK1 and PROK2 in WHO grade. (c) Expression of low and high concentrations of PROK1 and PROK2 in gender. (d) Expression of low and high concentrations of PROK1 and PROK2 in age. (e) Expression of low and high concentrations of PROK1 and PROK2 in IDH status. (f) Expression of low and high concentrations of PROK1 and PROK2 in histological type. (g) Expression of low and high concentrations of PROK1 and PROK2 in 1p/19q codeletion.

**Figure 5:** PROK1 and PROK2 multivariate Cox analysis of forest plot. As tumor grade, age, IDH status, 1p/19q codeletion, and PROK1 and PROK2 expression are independent prognostic factors.

**Figure 6:** The proportion of 21 immune cells affected by the expression of PROK1 and PROK2. PROK1 and PROK2 had 21 TIICs (Th1 cells, NK CD 56bright cells, and Mast cells had significant difference in PROK1 and PROK2).

**Figure 7:** Expression difference of Pan cancer between PROK1 and PROK2. (a) The expression of PROK1 was significantly different in BLCA, BRCA, COAD, HNSC, KICH, KIRP, and PRAD (*P* < 0.001). (b) The expression of PROK2 was significantly different in BRCA, LIHC, LUAD, LUSC, and UCEC (*P* < 0.001).

**Figure 8:** Venn of prokineticins and hub genes. (a) The Venn intersection of PROK1 and PROK2 yields 21 DEGs. (b) Protein-protein interaction network of hub genes (enrichment *P* = 6.82e-09).

**Figure 9:** Heat map of correlation analysis between PROK1 and PROK2 and hub genes. Except for the nonsignificant correlation between GATA4 and PROK1, the remaining hub genes were significantly different for PROK1 (a) and PROK2 (b).

**Figure 10:** Enrichment plots from gene set enrichment analysis (GSEA). (a) GSEA results showing differential enrichment of genes with high PROK1 expression. (FCMR activation, initial triggering of complement, creation of C4 and C2 activators, CD22-mediated BCR regulation, and complement cascade). (b) GSEA results showing differential enrichment of genes with low PROK1 expression (cytoplasmic ribosomal proteins, ribosome, rRNA processing, eukaryotic translation initiation, and eukaryotic translation elongation). (c) GSEA results showing differential enrichment of genes with high PROK2 expression (scavenging of heme from plasma, CD22-mediated BCR regulation, creation of C4 and C2 activators, FCGR activation, and role of LAT2 NTAL lab on calcium mobilization). (d) GSEA results showing differential enrichment of genes with low PROK2 expression (ribosome, cytoplasmic ribosomal proteins, activation of the mRNA upon binding of the cap binding complex and eifs and subsequent binding to 43 s, rRNA modification in the nucleus and cytosol, and mRNA splicing minor pathway).

**Table 1:** Clinical baseline data of different concentrations of PROK1 and PROK2.

Characteristic	Low expression of PROK1	High expression of PROK1	*P*	Low expression of PROK2	High expression of PROK2	*P*
*N*	264	264		264	264	
WHO grade			**0.047**			0.974
G2	123 (26.3%)	101 (21.6%)		111 (23.8%)	113 (24.2%)	
G3	110 (23.6%)	133 (28.5%)		119 (25.5%)	124 (26.6%)	
Gender			1			0.08
Female	119 (22.5%)	120 (22.7%)		109 (20.6%)	130 (24.6%)	
Male	145 (27.5%)	144 (27.3%)		155 (29.4%)	134 (25.4%)	
Age, meidan (IQR)	38 (31, 48)	43.5 (33, 55)	**< 0.001**	41 (33, 50)	39 (31.75, 55.25)	0.613

**Table 2:** PROK1 and PROK2 are associated with hub genes, Pearson's coefficient, and *P* values.

Hub genes	PROK1		PROK2	
	Pearson	*P*	Pearson	*P*
HOXC10	0.130	0.003	0.277	<0.001
HOXD13	0.104	0.017	0.184	<0.001
SOX4	-0.093	0.033	-0.264	<0.001
GATA4	0.061	0.158	0.235	<0.001
HOXA9	0.128	0.003	0.203	<0.001

## Data Availability

The datasets used and/or analyzed during the current study are available from the corresponding author on reasonable request.
